The article "miR-1226-3p Promotes eNOS Expression of Pulmonary Arterial Endothelial Cells to Mitigate Hypertension in Rats via Targeting Profilin-1" was retracted in 2024. Reasons: signs of a paper mill; suspected computer-generated content; unreliable results or conclusions; concerns about the data.

# miR-1226-3p Promotes eNOS Expression of Pulmonary Arterial Endothelial Cells to Mitigate Hypertension in Rats via Targeting Profilin-1

**DOI:** 10.1155/2021/1724722

**Published:** 2021-11-03

**Authors:** Jie Jian, Liang Xia

**Affiliations:** ^1^Department of Cardiac Surgery, Guangdong Cardiovascular Institute, Guangdong Provincial People's Hospital, Guangdong Academy of Medical Sciences, Guangzhou 51000, Guangdong Province, China; ^2^Department of Critical Care Medicine, The First Affiliated Hospital of Chongqing Medical University, 400016 Chongqing, China

## Abstract

In pulmonary arterial hypertension (PAH), microRNAs (miRNAs) are related with dysfunction of pulmonary arterial endothelial cells. miR-1226-3p was found to be downregulated in the serum of PAH patients, while few studies have illustrated the regulation mechanism of miR-1226-3p on PAH. In this study, we aimed to systematically investigate the role of miR-1226-3p in PAH. Sprague-Dawley (SD) rats were treated with monocrotaline (MCT) to establish the PAH models. The right ventricular systolic pressure (RVSP), ratio of the right ventricle to the left ventricle with septum (RV/(LV+S) ratio), and nitric oxide (NO) content were used to reflect the symptom of the rats. The rat models were used to observe the regulation mechanism of miR-1226-3p on PAH, and dual-luciferase reporter assay was used to verify the binding effect of miR-1226-3p to Pfn1. Besides, the qRT-PCR and western blot were used to measure the expression levels of miR-1226-3p and some keys proteins such as eNOS and Pfn1, respectively. The results showed that the PAH models were established successfully. The RVSP levels and the RV/(LV+S) ratio of the PAH rats were higher than those indexes in normal rats, while the NO content showed the opposite trends. Besides, the decreased miR-1226-3p and eNOS were, respectively, found in the PAH rats and rPAECs, and overexpressed miR-1226-3p could reverse the disadvantages of the PAH rats including increased RVSP, high RV/(LV+S) ratio, and decreased NO content. Furthermore, miR-1226-3p could directly target the 3′-UTR of Profilin-1 (Pfn1). Overexpressed Pfn1 led to decreased eNOS, while miR-1226-3p could partly inhibit the expression of Pfn1 and increase the expression level of eNOS in rPAECs. In summary, this study suggests miR-1226-3p as a protector to increase eNOS, improve NO content in rPAECs of the PAH rats via targeting Pfn, and finally protect the rats from the injury induced by PAH.

## 1. Introduction

Pulmonary arterial hypertension (PAH) is characterized by increased pulmonary vascular resistance, right heart failure, and high mortality [1, 2]. Even with the current medical conditions, the 5-year survival of patients remains unsatisfactory [3, 4]. Furthermore, the pathological changes of the tissues such as inflammation and pulmonary vasoconstriction had already happened by the time patients were diagnosed with PAH. As a potential interventional point, consideration has been given to the increased arterial pressure induced by nitric oxide (NO) deficiency in endothelial cells, which is a hallmark event of PAH. The synthesis dysfunction of vasodilator NO is well considered a major reason of PAH [5, 6]. Abnormal expression and dysfunction of the endothelial NO synthase (eNOS) in the human pulmonary arterial endothelial cells (HPAECs) leads to decreased NO content and thus contributes to the development and progression of PAH [7, 8].

MicroRNAs (miRNAs) are small, highly conserved, noncoding RNA molecules involved in regulating gene expression. They target mRNA molecules for cleavage or translational repression, resulting in the degradation of mRNA and/or the inhibition of mRNA translation [9, 10]. Abnormal expression of miRNAs is implicated in several diseases including some cancers and multiple cardiovascular diseases. Moreover, modulating the expression level of some factors has been thought as a promising therapeutic strategy of miRNAs in clinical intervention [11, 12]. Consequently, highlighting the usefulness of miRNAs as diagnostic and prognostic targets is necessary [13]. In PAH, miRNAs are related with dysfunction of pulmonary arterial endothelial cells [14, 15]. One study has found that miR-1226-3p was downregulated in the serum of patients with PAH, while few studies have illustrated the regulation mechanism of miR-1226-3p on PAH [16].

Recently, profilin 1(Pfn1), a regulator of actin dynamics, emerged as a potential new player in the field. Pfn1 is abundant in stable atherosclerotic plaques and in thrombi extracted from infarct-related arteries in patients with acute myocardial infarction. In this study, the expression level of miR-1226-3p in a rat model was determined to analyze its effect in PAH pathologies. Furthermore, the potential target gene of miR-1226-3p was investigated to illustrate its regulation mechanism on PAH.

## 2. Materials and Methods

### 2.1. Animal Models

50 male Sprague-Dawley (SD) rats (weight: 210 ± 10 g, average age: 6-8weeks) were purchased from Betterbiotechnology Co., Ltd. (Nanjing, China). All animals were given freedom to obtain food and water at any time. The rats (*n* = 20) were randomly divided into the control and PAH groups. Monocrotaline (MCT) was purchased from MedChem Express (New Jersey, USA), and the rats in the PAH groups were injected with MCT at 60 mg/kg to establish the pulmonary hypertension models, while rats in the control group were injected with normal saline.

Rats (*n* = 30) were randomly divided into three groups, including a PAH+saline group, a PAH+miR-NC group, and a PAH+miR-1226-3p group. In addition, at the time points of 48 hours before MCT treatment and 7 and 14 days after MCT treatment, the rats in the MCT+miR-1226-3p group and in the MCT-miR-NC group were infected with miR-1226-3p overexpressed lentivirus and negative control miRNA (miR-NC) lentivirus (2 × 10^8^ TU/ml per rat), respectively. All lentivirus were constructed by Hanbio Biotechnology Co., Ltd. (Shanghai, China).

After 21 days of MCT treatment, rats were anesthetized and then used to measure the hemodynamics. The biological data acquisition and analysis system (BL-420s, Techman Sorfware Co., Ltd., Chengdu, China) was used to measure the right ventricular systolic pressure (RVSP) and ratio of the right ventricle to the left ventricle with septum (RV/(LV+S) ratio) of rats. After that, the lung tissues of rats were collected for the following experiments.

### 2.2. Measurement of the Level of NO

The level of NO in the homogenate of lung tissues was determined as described previously. NO was detected with a Sievers chemiluminescence nitric oxide analyzer (Model 280; Sievers, Boulder, USA). Standard curves with NaNO_3_ were performed daily.

### 2.3. Cells Culture

The pulmonary arteries obtained from normal rats were used to isolate the rat arterial endothelial cells (rPAECs). The cells were cultured in DMEM (Thermo Fisher Scientific, Massachusetts, USA) which included 10% fetal bovine serum (FBS, Hyclone, South Logan, UT, USA). All cells were incubated in incubator at 37°C.

### 2.4. Cell Transfection

When the rRAECs were cultured at 70% confluence, the miR-1226-3p mimic, miR-NC or Pfn1 overexpression plasmid (pCMV-Pfn1) were transfected into cells with Lipofectamine 2000 (Invitogen, California, USA), and then, cells were incubated in incubator at 37°C for 48 h. In addition, all of miR-1226-3p mimic, miR-NC, and pCMV-Pfn1 were purchased from Beijing Generay Biotech Co., Ltd (Beijing, China).

### 2.5. qRT-PCR

Total RNAs of the tissues or cells were extracted by a TRIzol reagent. After that, the extracts were transcribed into cDNA by a PrimeScript® RT reagent Kit (Thermo Fisher, Massachusetts, USA). The primers of miR-1226-3p were synthesized and purified by Synbio Technology (Suzhou, China). According to the operation instruction of the KAPA qRT-PCR kit (Sigma-Aldrich, Missouri, USA), the reaction systems (10 *μ*l) were prepared for qRT-PCR, and the reaction conditions included predenaturation at 95°C for 30 s, 95°C for 5 s, and 60°C for 30s for a total of 40 cycles. U6 was used as the control of miR-1226-3p. The sequences of forward and reverse primer of miR-612 and U6 have been shown in Table 1.

### 2.6. Western Blot

The total protein of the tissues or cells were extracted by RIPA buffer (containing 1% PMSF for keep stability of proteins), and the concentration of total proteins was measured by BCA protein assay kit (Beyotime, Shanghai, China). All proteins were separated by 10% SDS-PAGE, and then, they were transferred from SDS-PAGE onto the PVDF membranes. After that, the nonfat milk with concentration at 5% was used to block membranes for 1 hour, and then, the membranes were incubated with the primary antibodies of target proteins at 4°C overnight, and the *β*-actin was used for quantification of target proteins. After washing three times with TBST, the membranes were incubated with the secondary antibodies for 1.5 hours at 25°C. Finally, a chemiluminescence detection system was used to observe protein expression level.

### 2.7. Dual-Luciferase Reporter Assay

The 3′-UTR fragments of Pfn1 and the mutant one were synthesized and inserted into the pmirGLO luciferase reporter vector (Promega, Wisconsin, USA). The reporter constructs were named as Pfn1-Wt and Pfn1-Mut, respectively. After that, the vectors of Pfn1-Wt and Pfn1-Mut were cotransfected into 293T cells with miR-1226-3p mimic or miR-NC, respectively. In addition, both miR-1226-3p mimic and miR-NC were purchased from Beijing Generay Biotech Co., Ltd. (Beijing, China).

### 2.8. In Vivo Experiment

Rats (*n* = 30) were randomly divide into three groups, including a PAH+saline group, a PAH+miR-NC group, and a PAH+miR-1226-3p group. In addition, at the time points of 48 hours before MCT treatment and 7 and 14 days after MCT treatment, the rats in the MCT+miR-1226-3p group and in the MCT-miR-NC group were infected with miR-1226-3p overexpressed lentivirus and negative control miRNA (miR-NC) lentivirus (2 × 10^8^ TU/ml per rat), respectively. All lentivirus were constructed by Hanbio Biotechnology Co., Ltd. (Shanghai, China).

After 21 days of MCT treatment, rats were anesthetized and then used to measure the hemodynamics. The biological data acquisition and analysis system (BL-420s, Techman Sorfware Co., Ltd., Chengdu, China) was used to measure the right ventricular systolic pressure (RVSP) and ratio of the right ventricle to the left ventricle with septum (RV/(LV+S) ratio) of rats. After that, the lung tissues of rats were collected for following experiments.

### 2.9. Statistical Analysis

All the experiments were performed at least three times, and the data were analyzed by SPSS 20.0, and the figures were charted by GraphPad Prism 8.0. The difference between the groups was calculated through Chi-squared test or ANOVA with Tukey's post hoc test. *P* < 0.05 means that it is statistically significant between two groups.

## 3. Results

### 3.1. The PAH Rat Models Were Established Successfully

To verified the utilizability of models after treating with MCT, the RVSP level and RV/(LV+S) ratio of the rats were detected. The results showed that the RVSP level and RV/(LV+S) ratio of the PAH rats were significantly higher than those indexes in the rats injected with normal saline (Figures 1(a) and 1(b), *P* < 0.05). Besides, it was observed that the content of NO in the lung tissue of the PAH rats significantly decreased compared with the normal rats (Figure 2(b), *P* < 0.05).

### 3.2. Decreased miR-1226-3p and Downregulated eNOS Were Observed in the Lungs of the PAH Rats and rPAECs, Respectively

To analyze the connection between miR-1226-3p and PAH, qRT-PCR was used to measure the expression level of miR-1226-3p in the lung tissues of the PAH rats. The results showed that miR-1226-3p was significantly downregulated in lungs of the PAH rats (Figure 2(a), *P* < 0.05). Besides, overexpressed miR-1226-3p increased the expression level of eNOS in rPAECs (Figures 2(c) and 2(d), *P* < 0.05).

### 3.3. miR-1226-3p Can Directly Target the 3′-UTR of Pfn1

To make sure the regulation mechanism of miR-1226-3p on PAH, the miRWalk, an online database, was used to predict the downstream targets of miR-1226-3p. The results showed that Pfn1 was one of potential factors, which had low binding energy with miR-1226-3p compared with the most of others. Based on this, dual-luciferase reporter assay was used to further confirm the accuracy of the forecast results. The results showed that miR-1226-3p can directly target the 3′-UTR of Pfn1-wt and inactivate the luciferase activity of the Pfn1-wt rather than Pfn1-mut (Figure 3(a), *P* < 0.05). Besides, the significantly increased expression level of BNF1 was observed in the rRAECs when miR-1226-3p was downregulated (Figures 3(b) and 3(c), *P* < 0.05).

### 3.4. miR-1226-3p Upregulated eNOS via Inhibiting the Expression of Pfn1

To explore the relationship of miR-1226-3p and Pfn1, the miR-1226-3p mimic and Pfn1 were cotransfected into rRAECs, and western blot and qRT-PCR were used to observe the expression levels of Pfn1 and miR-1226-3p, respectively. The results showed that the Pfn1 inhibited the expression of eNOS in rRAECs, while miR-1226-3p could reverse this phenomenon (Figures 4(a)–4(d), *P* < 0.05).

### 3.5. miR-1226-3p Alleviated the Symptom of the PAH Rats

To verify the function of miR-1226-3p in protecting rats away from the injury induced by PAH, the lentivirus of miR-1226-3p were used to infect the PAH rats, and the RVSP level, RV/(LV+S) ratio, and NO content of the PAH rats were detected. The results showed that the RVSP level and RV/(LV+S) ratios significantly decreased in the PAH rats infected with lentivirus of miR-1226-3p compared with the PAH rats infected with lentivirus of miR-NC (Figures 5(a) and 5(b), *P* < 0.05). Besides, the NO content in lung tissues of the PAH rats infected with lentivirus of miR-1226-3p increased significantly (Figure 5(c), *P* < 0.05).

## 4. Discussion

It is confirmed that the increased NO content in the blood is a pathway of regulating blood pressure in mammals, which could prevent and improve the symptom of PAH [17]. One study has indicated that the expression level of miR-1226-3p is significantly decreased in the peripheral blood of patients with PAH [16]. Therefore, this study has focused on the connection between miR-1226-3p and PAH. We demonstrated that the expression level of miR-1226-3p decreased significantly in lungs of the PAH rats, and overexpressed miR-1226-3p could alleviate the symptom of the PAH rats including high RVSP level, high RV/(LV+S) ratio, and low NO content in the lung tissues. It was found that the synthesis progression of NO in the blood of the PAH rats could be attenuated when the rats were treated with MCT, and the level of miR-1226-3p could influence the protein level of eNOS in rPAECs. Furthermore, we confirmed that miR-1226-3p directly targeted the 3′-UTR of Pfn1 which was an upstream regulator of eNOS, and miR-1226p reversed the phenomenon of decreased eNOS in rPAECs induced by overexpressed Pfn1. Those observations suggest that miR-1226-3p could alleviate the symptoms of the PAH rats through activating the eNOS/NO pathway via targeting Pfn1.

MCT exposure is a common method used in rats to establish the models to imitate the symptoms of the patients with PAH [18, 19]. In this study, MCT was also used to induce to the formation of PAH in normal rats, and the pathological changes of the PAH rats proved by several experiments, including the RVSP level and RV/(LV+S) ratio, suggested that the models were established successfully. Based on this, we found that miR-1226-3p was downregulated in the lung tissues of the rats treated with MCT, which suggests that miR-1226-3p may have a potential connection with the PAH. Besides, it was also captured that overexpressed miR-1226-3p could diminish the alterations of the PVSP level, RV/(LV+S) ratio, and NO content in the lung tissues of the PAH rats induced by MCT treatment. Those observations suggest that the deficiency of miR-1226-3p, and eNOS is a potential reason to contribute the formation of PAH in the rats treated with MCT.

There are many factors causing pulmonary hypertension, including hypoxia, oxidative stress, and the pathological changes in pulmonary vascular structure [20–22]. As a key substance, NO is synthesized by eNOS and can improve the symptom of PAH in patients via alleviating the pressure of arterial artery [23]. In the PAH rats, the decreased NO level in lung tissues of the PAH rats was observed, and the expression level of eNOS was also found to be downregulated in rPAECs, significantly. Those observations support that eNOS deficiency and decrease of NO may be the major reasons in formation of PAH.

Recently, some studies have indicated that eNOS is downregulated in human pulmonary artery endothelial cells, and its expression level is modulated by many factors [24]. The functions of regulating in translation of mRNAs is a common mechanism of miRNAs in taking parts in cellular life activities, and some miRNAs can directly involve in the progression of hypertension via mediating the expression level of eNOS in vascular endothelial cells [25, 26]. In this study, we found that eNOS was upregualated in rRAECs when miR-1226-3p was overexpressed. At present, few studies have illustrated the regular mechanism between miR-1226-3p and eNOS. For miR-1226-3p, it has been found to take a part in regulations of several diseases via targeting the key factors in pathways [27]. A growing amount of data associate Pfn 1, a protein crucial for cell biology, with the pathogenesis of coronary artery disease. It is increasingly clear that Pfn1 functions far beyond its well-known role as an actin dynamic regulator. In this study, Pfn1 was predicted as a potential target of miR-1226-3p by miRWalk, and miR-1226-3p could reduce the luciferase activity of Pnf1 via directly targeting with 3′-UTR of Pnf1. Pfn1 has connected with many diseases of human, and its overexpression contributes to the decreased eNOS in the vascular endothelial cell [28, 29]. We also confirmed that overexpressed Pfn1 induced the downregulation of eNOS, while miR-1226-3p could partly reverse the effect of Pfn1 on the expression of eNOS.

## 5. Conclusion

In summary, our study suggests that miR-1226-3p plays a protector role in alleviating the symptoms of the PAH rats though promoting the eNOS expression in HPAECs via targeting Pfn1.

## Figures and Tables

**Figure 1:** The PAH rats were established successfully. (a) The RVSP level of the rats. (b) The RV/(LV+S) ratio of the rats. Statistical analysis is by one-way ANOVA with Turkey's post hoc analysis. ^∗^*P* < 0.05.

**Figure 2:** miR-1226-3p was downregulated in the lung tissues of the PAH rats. The NO content in the lung tissues of the PAH rats decreased significantly, and eNOS was upregulated in rPAECs when miR-1226-3p was overexpressed. (a) The relative expression level of miR-1226-3p in the lung tissue of the PAH rats. (b) The NO level in the lung tissue of the PAH rats. (c, d) The relative protein expression level of eNOS in rPAECs. ^∗^*P* < 0.05.

**Figure 3:** miR-1226-3p directly targeted the 3′-URT of Pfn1, and overexpressed miR-1226-3p inhibits the expression of Pfn1. (a) miR-1226-3p reduced the luciferase activity of Pfn1-wt. (b, c) The relative protein expression level of Pfn1 in HPAECs transfected with miR-1226-3p mimic. ^∗^*P* < 0.05.

**Figure 4:** Pfn1 inhibited the expression of eNOS, while miR-1226-3p reversed the effect of Pfn1 on eNOS. (a) The relative expression level of miR-1226-3p. (b–d) The relative protein expression levels of PFN1 and eNOS. ^∗^*P* < 0.05.

**Figure 5:** miR-1226-3p protected the PAH rats away from the injury induced by MCT. (a) The RVSP level of the PAH rats in the groups of saline, miR-NC, and miR-1226-3p. (b) The RV/(LV+S) ratio of the PAH rats in the groups of saline, miR-NC, and miR-1226-3p. (c) The NO level of the PAH rats in the groups of saline, miR-NC, and miR-1226-3p. ^∗^*P* < 0.05.

**Table 1:** Primer sequence of miR-1226-3p and U6.

Name of primer	Sequences
miR-1226-3p-F	5′-GCGGCTCACCAGCCCTGTGT-3′
miR-1226-3p-R	5′-CAGCCACAAAAGAGCACAAT-3′
U6-F	5′-CTCGCTTCGGCAGCACA-3′
U6-R	5′-AACGCTTCACGAATTTGCGT-3′

## Data Availability

The authors confirm that the data supporting the findings of this study are available within the article.
